# A Meta-Analysis of the Differences in Serum Lipid Levels between Pregnant Women with Hypertensive Disorder Complicating Pregnancy and Nonhypertensive Disorder Complicating Pregnancy

**DOI:** 10.1155/2022/8974924

**Published:** 2022-10-03

**Authors:** Yong Zhang, Yonghong Pei, Na Li

**Affiliations:** Department of Obstetrics and Gynecology, Jinling Hospital, Clinical School of Medical College, Nanjing University, Nanjing, China

## Abstract

**Background:**

Although a lot of research work has been done on the etiology and pathogenesis of hypertensive disorder complicating pregnancy at home and abroad, the exact etiology and pathogenesis of the disease are still uncertain so far.

**Aims:**

Systematic review of meta-analysis of differences in serum lipid levels between pregnant women with hypertensive disease complicated with pregnancy and nonhypertensive disease complicated with pregnancy.

**Materials and Methods:**

PubMed, Medline, Embase, Science Citation Index (SCI), Cochrane, Springer, CNKI, Wanfang, VIP, and other databases were used to retrieve published literature and evaluate the included literature according to the quality evaluation method of medical literature introduced by the Cochrane Collaboration. A systematic review of the included studies was performed by meta-analysis.

**Results:**

We included 9 articles that documented total bile acids and D-dimers. In the heterogeneity test (*P* < 0.05, *I*^2^ = 100% > 50%), it was considered that the study was heterogeneous, so sensitivity analysis was used, the fixed-effect model was replaced, and the results were not significantly different after each item was excluded. Reliably, the difference was statistically significant (*Z* = 7.32, *P* < 0.001). In the TG metaheterogeneity test,*P* < 0.05,*I*^2^ = 99% > 50%, to explore the source of heterogeneity and conduct sensitivity analysis and switch to fixed-effect model, the difference was not statistically significant (*P* > 0.05). There was no significant difference in TC between hypertensive disorder complicating pregnancy and nonhypertensive disorder complicating pregnancy (*P* > 0.001).

**Conclusion:**

D-dimer, total bile acids, and glycopyrrolate were highly expressed in the sera of pregnant women with hypertensive disorder complicating pregnancy dyslipidemia.

## 1. Introduction

Hypertensive disorder of pregnancy (HDCP) is a unique pregnancy disorder, which is a group of diseases coexisting with pregnancy and hypertension [1]. Although a lot of research work has been done at home and abroad on the etiology and pathogenesis of the disease, the exact etiology and pathogenesis of the disease are still uncertain so far [2]. Pregnancy is a special period in which the metabolic function of women changes, and during the first trimester of pregnancy, lipids are elevated due to increased lipogenesis and lipolytic inhibition [3]. In addition, increased lipolysis and increased fatty acid content can be expected in the middle of pregnancy [4]. Maternal energy metabolism in midpregnancy is directed towards lipolysis, which leads to increased levels of circulating fatty acids [5]. In late pregnancy, enhanced lipolytic activity in maternal adipose tissue leads to maternal hyperlipidemia.

These changes in lipid metabolism indicate physiological adaptations in the mother's body that result in the conversion of glucose metabolism to lipid metabolism, which in turn provides nutrition for fetal development [6]. Several studies have shown that blood lipids in pregnant women begin to rise during pregnancy at 13 weeks of gestation, reach a peak around 28 weeks of gestation, and decline significantly within 1 day after delivery until they gradually return to normal in the late puerperium, although some pregnant women experience prolonged hyperlipidemia for several years after delivery [7]. High levels of total cholesterol (TC), triglycerides (TG), and low-density lipoprotein (LDL) and/or low high-density lipoprotein (HDL) levels are risk factors for arteriosclerosis [8]. The early stages of atherosclerosis are the deposition of lipid-rich macrophages in the vessel wall, and the exact pathophysiological mechanisms are not known [9]. We hypothesize that on the one hand, the distribution of atherosclerotic lipids increases the risk of endothelial damage via oxidative stress mechanisms in the arterial vessel wall. On the other hand, the increased peroxidation of these elevated plasma lipids leads to enhanced oxidative stress through the progressive production of free radicals and lipid peroxides [10]. Lipid peroxides are toxic compounds that may damage endothelial cells, and these contribute to gestational hypertension and/or prehypertension [11]. The exact pathophysiology of HDCP remains to be elucidated, but the current hypothesis is that the symptoms of HDCP are caused by endothelial dysfunction associated with placental hypoxia, which leads to local inflammation and oxidative stress with acute atherosclerosis of the placental spiral arteries [12]. Scholars believe that the accumulation of large amounts of cholesterol-rich particles contributes to the formation of atherosclerosis; however, it may also be caused by triglyceride-rich particulate matter [13]. Studies have shown that prenatal serum TG and free fatty acid concentrations increase approximately 2-fold in women with HDCP relative to pregnant women with simple pregnancy, with no effect on total cholesterol, HDL, and LDL [14].

Meta-analysis is defined as a quantitative review that specifically includes asking research questions, searching relevant literature, developing inclusion and exclusion criteria for the literature, summarizing basic information, synthesizing the analysis, and reporting the results [15]. Therefore, meta-analysis is more likely to present a convincing evidence-based basis than a general review. In our study, we collected the published literature on the differences in serum lipid levels between hypertensive disorder complicating pregnancy and nonhypertensive disorder complicating pregnancy in recent years at home and abroad and performed meta-analysis. The study was conducted in order to provide evidence-based medical evidence for clinical treatment.

## 2. Material and Methods

### 2.1. Diagnostic Criteria

According to the International Society for the Study of Hypertension in Pregnancy (ISSHP) guidelines for the classification, diagnosis, and management of hypertension [16], gestational hypertension is defined as systolic blood pressure ≥ 140 mmHg and/or diastolic blood pressure ≥ 90 mmHg measured on at least 2 occasions on the same arm. It is recommended to use an electronic sphygmomanometer to measure blood pressure, and the cuff size is required to be moderate. Severe blood pressure elevations (systolic blood pressure ≥ 160 mmHg and/or diastolic blood pressure ≥ 110 mmHg) should be confirmed by repeat measurement within 15 minutes, and mild blood pressure increases should be repeated within 4-6 hours. Urinary protein is no longer required for the diagnosis of preeclampsia.

### 2.2. Exclusion Criteria

Inclusion criteria were as follows: (1) the types of published literatures must be collected based on RCT trials regardless of whether they are blinded or not, and the languages are limited to Chinese and English; domestic and foreign published literature between January 1, 2010, and July 14, 2022; and the content of which involves risk factors related to the development of hypertensive disorder complicating pregnancy; (2) hypertensive disorder complicating The main risk factors commonly found in clinical practice for pregnancy include (1) maternal age, (2) BMI at the time of first delivery, (3) history of preeclampsia, (4) psychosocial stress, (5) first pregnancy, (6) history of chronic hypertension, (7) nutritional deficiency, (8) diabetes mellitus, (9) literacy level, and (10) family history of hypertension in pregnant women (mother or sister); (3) independent case-control studies; and (4) the included literature data can extracted complete experimental data.

Exclusion criteria were as follows: (1) exclusion of non-case-control study literature such as reviews, conference papers, lectures, and abstracts; (2) literature with incomplete access to data information; (3) literature with too low a quality rating; (4) literature with noncompliant study methods (not case-control studies or cohort studies); and (5) studies without a control group and studies in which the control group was nonconventional treatment. For repeated studies by the same author or the same unit, if two papers reported overlapping data, then the one with the larger patient sample size was selected and the one with the smaller sample size was excluded; if both the sample size and the observed indicators were consistent, the one with the higher published journal score was selected.

### 2.3. Search Strategy

According to the literature search requirements of the Cochrane Collaboration, online searches were conducted through PubMed, Medline, Embase, Science Citation Index (SCI), Cochrane, Springer, CNKI, Wanfang, and Vipul databases on hypertensive disorder after 2010. We searched the references of the included literature and collected as much as possible comprehensive literature on this study in Chinese and English. The Chinese search terms were as follows: (1) disease type: “hypertensive disorder complicating pregnancy” or “eclampsia” or “hyperemesis gravidarum”; (2) relevant index: “serum lipids”; and (3) study method: “randomized control” or “randomized”. The English search terms were retrieved by combining the corresponding subject terms with key words according to the characteristics of each database, and the duplicate literature was excluded. In English, (1) disease type: “gestational hyHDCPrtension” or “eclampsia” or “pregnancy-induced hyHDCPrtension”; (2) intervention: “serum lipids”; and (3) study method: “ROT “OR “Randomized control”.

### 2.4. Literature Screening and Quality Evaluation

All the collected literature was screened by two researchers, and the literature was screened in strict accordance with the established exclusion and inclusion criteria, and data were extracted from the final screened literature. Available data information on (i) maternal age, (ii) BMI at first obstetric examination, (iii) history of pre-eclampsia, (iv) family history of hypertension, (v) history of chronic hypertension, (vi) first pregnancy, (vii) nutritional deficiency, (viii) diabetes mellitus, (ix) literacy, and (x) psychosocial stress was extracted from the literature meeting the criteria for inclusion in the study.

### 2.5. Extraction of Information for Inclusion in the Literature

After evaluating the quality of the literature, relevant information for use as a systematic review needs to be extracted from the literature that meets the inclusion requirements and organized and entered into Excel to create a database. The main information includes the following: (i) general information, such as literature title, source, author, and publication date; (ii) study characteristics: study design protocol and quality, study site, characteristics of the study population, implementation methods, measures to prevent bias, etc.; and (iii) study results: main study results, outcome indicators, etc.

### 2.6. Statistical Analysis

Meta-analysis was performed using RevMan 5.3 statistical software. The ratio of ratios (OR) was used as the result of the representation of effect sizes of categorical variables. Heterogeneity between studies was analyzed by the *Q*-test, and if the final heterogeneity test result *P* was greater than 0.1, it indicated that the studies were homogeneous and a fixed-effect model should be used for comprehensive analysis; if *P* was less than 0.1, it indicated that the studies were not homogeneous. If there is heterogeneity among the studies, the heterogeneity is further analyzed quantitatively by calculating the value, and if *I*^2^ is less than 50%, then the fixed-effect model is selected; if the result is *P* ≥ 0.10 and *I*^2^≦50%, it means that there is no obvious heterogeneity among the observed groups, and the fixed-effect model is selected to describe the data; if the result of heterogeneity test is *P* < 0.10 and *I*^2^ > 50%, it means that heterogeneity exists among the groups The source of heterogeneity was examined, and the results were also subjected to subgroup analysis or sensitivity analysis, and the final homogeneity was used in a fixed-effect model, while the random-effects model was used to combine effect values for different qualities, and descriptive analysis was used for literature not suitable for inclusion in meta-analysis. Econometric information for the analysis of continuous variables was expressed using weighted mean differences (WMD) and their 95% confidence intervals, with differences considered statistically significant at *P* < 0.05.

## 3. Results

### 3.1. Literature Search Results

After database search, a total of 368 literatures related to hypertensive disorder complicating pregnancy were finally retrieved. Duplicate literatures from different databases were excluded. After reading the titles and abstracts of the literatures, 80 literatures that met the inclusion criteria were preliminarily screened. 71 literatures that did not meet the inclusion criteria were excluded, and 9 literatures were finally included.

### 3.2. Basic Information of Included Studies

A total of 9 literatures were included in our study, including a total of 1238 patients, the average age of the patients was 29.34 ± 3.25, and 9 literatures had clear diagnostic criteria (see Table 1).

### 3.3. Publication Bias in Meta-Analysis

Bias in meta-analysis includes publication bias, literature base bias, inclusion criteria bias, and English language bias, of which the most common bias is publication bias. Publication bias refers to the fact that a statistically significant study result is more likely to be reported and published than a negative result that is not statistically significant. In order to ensure the authenticity and reliability of meta-analysis findings, possible publication bias should be identified and evaluated. The identification methods of bias include sensitivity analysis, funnel plot, rank correlation test, and fail-safe number. In this paper, a funnel plot is used to assess publication bias. If the final graph is an inverted funnel shape, there is no publication bias; conversely, if the graph is incomplete or asymmetric, there is a possibility of publication bias. As the sample size increases and the standard error decreases, the results are concentrated in a narrower range in the upper part of the graph. Therefore, the presence or absence of publication bias can be visualized by a funnel plot.

### 3.4. Metasensitivity Analysis

In order to judge the stability of the obtained results, it is possible to observe whether and to what extent the results and heterogeneity change after changing some important factors affecting the results, such as inclusion and exclusion criteria, statistical methods (fixed-effect model or random-effects model), and the choice of effect size (O or RR). The purpose is to discover the main risk factors and causes of generation that affect the results of meta-analysis. If the results before and after sensitivity analysis do not differ significantly, it indicates that the results are more reliable; if the results before and after sensitivity analysis are inconsistent, caution should be exercised when interpreting the results and drawing conclusions, suggesting that there may be potential factors influencing the results and further research is needed to clarify them.

### 3.5. Metaheterogeneity Test and Model Analysis

In the test of heterogeneity in meta-analysis in this paper, the*Q*test was used to calculate the resultant*P*value, and if the *P* value was greater than 0.1, it indicated that the studies were homogeneous, and if the *P* value was less than 0.1, it indicated that the studies were heterogeneous, but the size of heterogeneity among the studies could not be determined. In this study, the calculated values were used to indicate the size of heterogeneity among the studies, and the *I*^2^ range was 0%-100%. If the *I*^2^ was less than 25%, the studies were mildly heterogeneous; if the *I*^2^ value was 25%-50%, the studies were moderately heterogeneous; if the *I*^2^ was greater than 50%, the studies were highly heterogeneous. A meta-analysis can be performed using fixed-effect models and random-effects models, and the final model to be used is subject to heterogeneity testing. If the results are homogeneous or heterogeneous, but the heterogeneity is small, the fixed-effect model is used. When the heterogeneity between studies is high, a random-effects model is used or only qualitative descriptive analysis or subgroup analysis is done without combining the results.

### 3.6. Hypertensive Disorder Complicating Pregnancy Meta-Analysis Results

On the test of heterogeneity, *P* < 0.05 and *I*^2^ = 100% > 50%, indicating significant heterogeneity in the included studies, sensitivity analysis was performed on the source of heterogeneity and *P* and *I*^2^ changed significantly, considering this article as a source of heterogeneity. After exclusion, heterogeneity was tested and *P* = 0.73 > 0.05. The study was homogeneous, so the fixed-effect model was used for analysis, and the results showed that *Z* = 12.46 and *P* > 0.05, and the difference was not statistically significant (see Figure 1).

### 3.7. Results of D-Dimer Meta-Analysis

The study reported D-dimers in patients with hypertensive disorder complicating pregnancy after treatment, and when there was heterogeneity between groups, the source of heterogeneity was examined (*P* = 0 < 0.05, *I*^2^ = 99%), and fixed-effect model was used for analysis. The results showed a statistically significant difference (*P* < 0.05) in the D-dimer scores of hypertensive disorder complicating pregnancy compared to nonhypertensive disorder complicating pregnancy (see Figure 2).

### 3.8. Results of Meta-Analysis of Total Bile Acids

Total bile acids were recorded in 9 of our included papers. On the test of heterogeneity (*P* < 0.05, *I*^2^ = 100% > 50%), the studies were considered to be heterogeneous; therefore, sensitivity analysis was used and the results were not significantly different after switching to the fixed-effect model as well as excluding each item was more plausible and the difference was statistically significant (*Z* = 7.32, *P* < 0.001) (see Figure 3).

### 3.9. Results of Glycopyrrolate Meta-Analysis

On the test of heterogeneity, *P* < 0.05 and *I*^2^ = 99% > 50%, the study was considered heterogeneous, so a random-effects model was used for analysis to explore the sources of heterogeneity, sensitivity analysis was performed, and switching to a fixed-effect model as well as excluding each item revealed a statistically significant decrease in heterogeneity (*Z* = 57.02, *P* < 0.001) (see Figure 4).

### 3.10. TG Meta-Analysis Results

On the test of heterogeneity, *P* < 0.05 and *I*^2^ = 99% > 50%, the study was considered heterogeneous, so a random-effects model was used for analysis to explore the sources of heterogeneity for sensitivity analysis, and the differences were not statistically significant (*P* > 0.05) when replaced with a fixed-effect model (see Figure 5).

### 3.11. Results of TC Meta-Analysis

The heterogeneity between studies was high (*P* < 0.05, *I*^2^ = 17% > 50%), and the random-effects model was used for analysis. The results showed that there was no statistically significant difference between the TC of hypertensive disorder complicating pregnancy compared with nonhypertensive disorder complicating pregnancy (*P* > 0.001) (see Figure 6).

## 4. Discussion

Hypertensive disorder complicating pregnancy has always been a hot topic and focus of investigation by experts and scholars in obstetrics, which involves the etiology, pathogenesis, risk factors, and prediction and prevention of the disease [17]. However, the exact etiology and pathogenesis of the disease have not yet “surfaced,” so in order to better predict and prevent the disease, the study of the common clinical risk factors for the disease is of great significance [18]. To date, there is a large literature on risk factors for HDCP, with a wide variety of literature and varying quality, but there is a lack of high-quality literature [19]. We read the literature on risk factors for this disease in the last decade, removed the dross and took the essence, and analyzed the most common clinical risk factors nowadays in an in-depth and systematic way [20].

The literature included in this study were all published case-control studies or cohort studies from the past 10 years or so at home and abroad, and each piece of literature was systematically scored by NOS evaluation criteria. Also, to avoid bias from those who selected the literature and those who evaluated the quality of the literature, two evaluators independently assessed the quality of the screened literature [21]. The included literature was clearer about the criteria for the diagnosis of HDCP and the factors exposed, so that bias caused by errors in the diagnosis of the disease and errors in the identification and determination of exposure factors was small [22]. For some reasons, more detailed, accurate, and high-quality literature could not be collected and included in the study, and significant confounding bias and any other bias in some of the literature that was included in the study were not excluded and systematically analyzed [23]. The meta-analysis in this study can obtain and further demonstrate the main risk factors for morning sickness and the strength of association with HDCP, which is more convincing than individual reviews or case-control or cohort studies and also provides valuable information for predicting and preventing morning sickness. According to the established inclusion and exclusion criteria, a total of 9 publications were finally included after a systematic and comprehensive search and rigorous quality evaluation. However, the quality of the included studies was assessed by the NOS evaluation criteria, and it was found that the quality of the studies in the literature varied, and those that were too low-quality were isolated [24]. Therefore, in order to obtain more accurate results with less bias, there is a need for higher quality case-control studies or cohort studies to be published in the literature [25]. Systematic reviews, like other studies, can have different biases at various stages of the study, which can bias the final comprehensive analysis from the true results [26]. The types of systematic review bias include publication bias, literature base bias, inclusion criteria bias, and English language bias. Literature base bias arises during the collection of the literature. Because there are no uniform criteria for inclusion in the literature, inclusion criterion bias may arise when researchers set their own inclusion criteria based on the content of the studies they need [27]. Since the literature collected was in English and Chinese, English bias could not be avoided [28]. In this paper, the research languages are limited to Chinese and English, and valuable research published in other languages was not retrieved and evaluated. However, publication bias is the most common and noteworthy issue in systematic reviews [29]. Although the literature related to risk factors for hyperemesis was collected as comprehensively as possible in this paper, there may still be underrepresentation due to the following reasons: the studies included in this paper were all published and there is a lack of evidence from unpublished studies and other nontraditional sources, which may exaggerate the strength of the association of certain risk factors due to the preponderance of “positive” results. The strength of the association of certain risk factors may be overstated because of the preponderance of “positive” results.

Under normal conditions, lipids circulating in the blood are usually lipoprotein complexes with high solubility, and during pregnancy, lipid levels may increase to some extent due to fetal growth and development [30]. Studies have shown that hypertensive disorder complicating pregnancy may be mainly caused by endothelial cell damage, and lipid peroxidation and inflammatory factors are the main factors causing endothelial cell damage, so dyslipidemia is associated with hypertensive disorder complicating D-dimer which is often used in clinical screening for thrombosis, and patients with hypertensive disorder complicating pregnancy have abnormal coagulation and present as a prethrombotic state [31]. Total bile acids and ethanoic acid are important substances produced by the liver during cholesterol degradation and are related to liver function. The results of this study showed that the levels of TG and TC, the lipid indexes of pregnant women with gestational hypertensive disease, were elevated compared with those of normal pregnant women, suggesting that gestational hypertensive disease is associated with abnormal lipid metabolism and that early detection of early lipid levels can help guide early intervention of the disease [32]. In this study, the overall incidence of D-dimer, total bile acids, glycolic acid, and adverse pregnancy outcomes was higher in dyslipidemic pregnant women than in normal-lipidemic pregnant women, and there was a correlation between lipid indices and D-dimer, total bile acids, and glycolic acid [33]. Studies have shown that abnormal lipid metabolism in early pregnancy increases the incidence of hypertensive disorder complicating pregnancy and adverse pregnancy outcomes, which is partially consistent with the results of this study [34]. It is suggested that high expression of D-dimer, total bile acids, and glycolic acid may be associated with hypertensive disorder complicating pregnancy maternal lipid energy and the development and progression of dyslipidemia. Close monitoring of serum D-dimer, total bile acids, glycolic acid, and lipid levels in pregnant women with hypertensive disorder complicating pregnancy in clinical practice may be important to ensure good pregnancy outcome and achieve eugenics [35].

The literatures included in our study are all case-control studies, which have certain shortcomings, which may come from the quality and quantity of literatures included in the study, as well as various biases that may appear in the research process. There are many risk factors related to PIH in the current research, but there are no systematic case-control studies and cohort studies. And some related factors are less likely to appear clinically. In addition, the results of systematic reviews are not static, because they are only the results of comprehensive analysis of existing data. Therefore, updated high-quality domestic and foreign research literature should be continuously searched, and new information should be updated and supplemented in time, so that the meta-analysis is more complete and the results are more convincing, providing a stronger evidence-based basis for the prediction and prevention of HDCP.

In conclusion, D-dimer, total bile acids, and glycopyrrolate were highly expressed in the sera of pregnant women with hypertensive disorder complicating pregnancy dyslipidemia.

## Figures and Tables

**Figure 1:** Hypertensive disorder complicating pregnancy meta-analysis of the number of cases.

**Figure 2:** D-dimer meta-analysis.

**Figure 3:** Total bile acid meta-analysis.

**Figure 4:** Glycopyrrolate meta-analysis.

**Figure 5:** TG meta-analysis.

**Figure 6:** TC meta-analysis.

**Table 1:** Basic characteristics of the included literature.

Author	Year of publication	Research site	Sample size	Age (years)
Ashraf Direkvand-Moghadam	2012	Iran	52	26.78 ± 3.32
Amal K. Suleiman	2014	Jordan	184	31.27 ± 4.22
Zou Lu	2015	China	150	33.78 ± 1.69
Zheng Jun	2019	China	102	23.74 ± 5.65
Standan	2017	China	40	29.34 ± 3.25
LCY Poon	2021	U.K.	305	29.52 ± 2.37
Wu Yan	2019	China	105	32.34 ± 3.25
Liu Zhong	2021	China	120	27.63 ± 1.32
Zhu Huifen	2012	China	180	31.93 ± 6.16

## Data Availability

The datasets generated during and/or analyzed during the current study are available from the corresponding author on reasonable request.
